# Comparison of Efficacy and Safety of Recombinant Human Prourokinase and Alteplase in the Treatment of STEMI and Analysis of Influencing Factors of Efficacy

**DOI:** 10.1155/2021/6702965

**Published:** 2021-09-06

**Authors:** Yizhou Liu, Yulin Yang, Ying Li, Xiaoqing Peng

**Affiliations:** ^1^The Affiliated Nanhua Hospital, Department of Cardiology, Hengyang Medical School, University of South China, Hengyang, Hunan 421001, China; ^2^The Affiliated Nanhua Hospital, Department of Recovery from Anesthesia, Hengyang Medical School, University of South China, Hengyang, Hunan 421001, China; ^3^The Affiliated Nanhua Hospital, Department of Nursing Teaching and Research, Hengyang Medical School, University of South China, Hengyang, Hunan 421001, China

## Abstract

**Objective:**

To compare the efficacy and safety of recombinant human prourokinase (rhPro-UK) and alteplase for thrombolytic therapy in acute ST-segment elevation myocardial infarction (STEMI) and to analyze the related factors affecting efficacy.

**Methods:**

From January 2017 to December 2019, 100 patients diagnosed with STEMI were selected and randomly divided into the control group (*n* = 50) and the observation group (*n* = 50). Based on conventional treatments, the control group was treated with alteplase, and the observation group was treated with rhPro-UK, and both were treated for 7 days. After treatment, the vascular recanalization, left ventricular end-systolic diameter (LVESD), left ventricular end-diastolic diameter (LVEDD), and left ventricular ejection fraction (LVEF) were compared. The bleeding and major adverse cardiovascular events (MACE) were recorded in both groups. According to the patient's vascular recanalization, it was divided into two subgroups: recanalization group and occlusion group. Multiple logistic regression models were used to analyze the related factors that affect the efficacy.

**Results:**

The recanalization rate of the observation group (96.00%) was higher than that of the control group (84.00%) (*P* < 0.05). After treatment, LVDs and LVEDD in both groups were lower than those before treatment, and LVEF was higher than that before treatment. The LVDs and LVEDD in the observation group were lower than those in the control group, and the LVEF was higher than that in the control group (*P* < 0.05). The incidence of bleeding in the observation group (2.00%) was lower than that in the control group (12.00%), and the incidence of MACE (4.00%) was lower than that in the control group (16.00%) (*P* < 0.05). Univariate analysis showed that age, smoking history, diabetes history, myocardial infarction history, infarct location, and intravenous thrombolysis time were related to the efficacy after treatment (*P* < 0.05). Multivariate logistic analysis showed that age, history of diabetes, vascular infarction site, and venous thrombolysis time were independent influencing factors after treatment (*P* < 0.05).

**Conclusion:**

Both rhPro-UK and alteplase thrombolytic therapy can effectively recanalize blood vessels and improve the cardiac function of patients with STEMI. However, rhPro-UK has better effect than alteplase and is safer and worth promoting. The curative effect is related to age, diabetes history, vascular infarction site, and venous thrombolysis time.

## 1. Introduction

ST-segment elevation myocardial infarction (STEMI) refers to patients with coronary artery atherosclerosis and plaque shedding, resulting in blood vessel blockage, resulting in a decrease in the heart's own blood supply and leading to myocardial ischemic necrosis [1, 2]. STEMI has the characteristics of rapid onset, rapid development, and high mortality rate. Patients experience myocardial injury or even death in a short period of time, which seriously endangers people's lives and health [3, 4]. At present, intravenous thrombolysis and percutaneous coronary intervention (PCI) are the main treatments for reperfusion therapy. Although the emergency PCI technology and process have matured, there are still some patients who cannot receive PCI treatment in time, such as patients stuck in traffic jams, patients in remote areas, and patients with severe hemodynamic instability. Therefore, timing is critical for intravenous thrombolytic therapy [5, 6]. Alteplase is a second-generation thrombolytic drug that can specifically activate plasminogen in thrombus and has a good thrombolytic effect [7, 8]. Recombinant human prourokinase for injection (rhPro-UK) is a new generation of thrombolytic drugs and the precursor of urokinase, which can be gradually metabolized into urokinase to quickly dissolve thrombus and make blood vessels unobstructed [9, 10]. This study used thrombolysis in myocardial infarction (TIMI) blood flow classification to evaluate the recanalization rate and compared the efficacy and safety of rhPro-UK and alteplase thrombolysis in STEMI patients. The detailed information is as follows.

## 2. Materials and Methods

### 2.1. General Information

100 patients diagnosed with STEMI in our hospital from January 2017 to December 2019 were selected as the research objects. Among them, 59 were males and 41 were females, aged from 32 to 76 years old, with an average age of 54.86 ± 9.42 years. Inclusion criteria: all patients meeting the diagnostic criteria of STEMI in “ESC Guidelines for the management of acute myocardial infarction in patients presenting with ST-segment elevation” [11]; no surgical treatment such as PCI; age ≤80 years; and time from onset to thrombolysis ≤6 hours. Exclusion criteria: those with severe liver and kidney dysfunction; those with arrhythmia; those with antiplatelet and anticoagulation contraindications; those who are allergic to study drugs. All patients were divided into control group and observation group by random number table, with 50 cases in each group. Among them, there were 30 males in the control group and 20 females, aged from 32 to 74 years old, with an average age of 54.45 ± 9.84 years. In the observation group, there were 29 males and 21 females, aged from 34 to 76 years, with an average age of 55.14 ± 9.18 years. There was no statistical difference between the two groups in general information (*P* > 0.05), and they were comparable. This study was approved by the ethics committee of our hospital, and the patients and their family members gave informed consent and signed an informed consent form.

### 2.2. Research Methods

All patients received conventional treatment including the following: oxygen inhalation and ECG monitoring for all patients were performed, nitrate esters for crown expansion were used, *β*-receptor blockers were used to reduce heart rate, angiotensin-converting enzyme inhibitors were used to inhibit myocardial remodeling, unfractionated heparin was used before and after thrombolysis for anticoagulation, etc. The control group was given 0.9 mg/kg alteplase for injection (Boehringer Ingelheim, National Medicine Standard S20110051), of which 10% was injected intravenously within 1 minute, and the remaining amount was intravenously injected within 60 minutes. The observation group used rhPro-UK (Shanghai Tasly Pharmaceutical Co., Ltd., National Medicine Standard S20110003), first mixed with 20 mg rhPro-UK and 10 ml sodium chloride solution and then injected intravenously. After the bolus injection was completed in about 3 minutes, 30 mg rhPro-UK was mixed with 90 ml sodium chloride solution and then instilled intravenously, and the infusion was completed in about 30 minutes. Patients in both groups were treated for 7 days.

Patients in both groups underwent coronary angiography after treatment, and vascular recanalization was assessed according to TIMI blood flow classification. TIMI classification: grade 3 is complete recanalization, grade 2 is vascular recanalization, grade 0∼1 is occlusion, recanalization rate = (number of complete recanalization cases + number of vascular recanalization cases)/total number of cases × 100%. Before treatment and 7 days after treatment, the patient's left ventricular end-systolic diameter (LVDs), left ventricular end-diastolic diameter (LVEDD), and left ventricular ejection fraction (LVEF) were checked by echocardiography. The bleeding and major adverse cardiac events (MACE) within 7 days of the two groups were recorded. According to the recanalization of patients, they were divided into two subgroups: recanalization group and occlusion group. The patient's smoking history, drinking history, diabetes history, hypertension history, myocardial infarction history, family history of coronary heart disease, vascular infarction location, intravenous thrombolysis time, and other relevant clinical data were recorded.

### 2.3. Statistical Methods

The data analysis was processed by SPSS22.0 software; the result of measurement data analysis is shown as mean ± standard deviation (mean ± SD), and the result of pairwise comparison between groups was analyzed by *t* test. The enumeration data are expressed in %, and the *χ*^2^ test is used. Multivariate analysis adopts multiple logistic regression model. The test level is *α* = 0.05, and *P* < 0.05 indicates that the difference is statistically significant.

## 3. Results

### 3.1. Comparison of Vascular Recanalization between the Two Groups

The recanalization rate of blood vessels in the observation group (96.00%) was higher than that in the control group (84.00%), and the difference was statistically significant (*P* < 0.05), as shown in Table 1.

### 3.2. Comparison of Cardiac Function between the Two Groups before and after Treatment

After treatment, the two groups of LVDs and LVEDD were lower than those before treatment, LVEF was higher than that before treatment, and the observation groups' LVDs and LVEDD were lower than those in the control group, LVEF was higher than that in the control group, and the difference was statistically significant (*P* < 0.05), as shown in Table 2.

### 3.3. Comparison of Bleeding between the Two Groups

In the control group, there were 2 cases of gum bleeding, 2 cases of nasal mucosal bleeding, and 2 cases of gastrointestinal bleeding. One case of gum bleeding occurred in the observation group. The incidence of bleeding in the observation group (2.00%) was lower than that in the control group (12.00%), and the difference was statistically significant (*P* < 0.05), as shown in Table 3 and Figure 1.

### 3.4. Comparison of the Incidence of MACE between the Two Groups

In the control group, there were 3 cases of heart failure, 3 cases of angina, 1 case of arrhythmia, and 1 case of recurrent myocardial infarction. In the observation group, there was 1 case of angina pectoris and 1 case of arrhythmia occurred. The incidence of MACE in the observation group (4.00%) was lower than that in the control group (16.00%), and the difference was statistically significant (*P* < 0.05), as shown in Table 4 and Figure 2.

### 3.5. Single Factor Analysis Affecting the Efficacy of Patients after Treatment

Univariate analysis showed that age, history of smoking, history of diabetes, history of myocardial infarction, vascular infarction location, and intravenous thrombolysis time were the factors related to the efficacy of the patient after treatment (*P* < 0.05), as shown in Table 5.

### 3.6. Analysis of Multiple Factors Affecting the Efficacy of Patients after Treatment

Multivariate logistic analysis showed that age, diabetes history, vascular infarction location, and intravenous thrombolysis time were independent factors influencing the efficacy of patients after treatment (*P* < 0.05), as shown in Tables 6 and 7.

## 4. Discussion

STEMI is mainly caused by the occurrence of myocardial ischemia and necrosis due to the rupture and shedding of unstable plaques in the coronary arteries, which leads to obstruction of the coronary arteries. SETMI has a rapid onset, extremely rapid disease progression, and high mortality. It requires timely reperfusion therapy to dredge the occluded blood vessels. Compared with PCI, intravenous thrombolysis has the advantages of simplicity, convenience, and speed and can effectively improve the treatment effect of STEMI patients [12, 13].

The results of this study showed that the vascular recanalization rate of the observation group (96.00%) was higher than that of the control group (84.00%), and the LVDs and LVEDD of the two groups after treatment were lower than those before treatment, and the LVEF was higher than that before treatment. The LVDs and LVEDD of the observation group were both lower than those of the control group, and LVEF is higher than that in the control group. It shows that both rhPro-UK and alteplase can effectively recanalize the blood vessels in STEMI patients and improve the patient's cardiac function, but the effect of rhPro-UK is better than that of alteplase. The reason is that alteplase is a recombinant tissue-type plasminogen activator, which can selectively bind fibrin and convert plasminogen into plasmin to exert a thrombolytic effect [14], and rhPro-UK can dissolve fibrin by binding to the fibrin of the thrombus. Once a thrombus is formed in the blood circulation, it induces the binding of fibrin Y/E fragments to prourokinase, thus exerting a thrombolytic effect, and its specificity is stronger, and the results of the study showed that the incidence of bleeding in the observation group (2.00%) was lower than that of the control group (12.00%), and the incidence of MACE (4.00%) was lower than that of the control group (16.00%).

In this study, single factor analysis showed that age, history of smoking, history of diabetes, history of myocardial infarction, location of vascular infarction, and intravenous thrombolysis time are related to the therapeutic effect after treatment. Multivariate logistic analysis showed that age, diabetes history, vascular infarction location, and intravenous thrombolysis time were independent factors influencing the efficacy of the treatment. Due to the decline in physical functions of elderly patients, the inner wall of the blood vessel is aging, the elasticity of the blood vessel is changed, and the intima is rough and damaged, which affects the effect of thrombolysis. Patients with a history of diabetes can easily lead to vascular endothelial damage due to abnormal glucose and lipid metabolism and vascular circulation, which accelerates the development of arteriosclerosis and affects thrombolysis [15]. Since the anterior wall myocardial infarction is mostly the left main coronary artery, compared with the inferior wall myocardial infarction of the right coronary artery disease, its clinical symptoms are more serious, and the treatment time is faster, and the effect is better. Drug thrombolysis is generally effective within 2 hours, and it is not easy to cause complications, so timely thrombolysis is helpful to improve the recanalization rate of infarcted vessels [16, 17].

In summary, both rhPro-UK and alteplase can effectively recanalize the blood vessels and improve the heart function of patients with STEMI. But compared with alteplase, rhPro-UK has better curative effect and higher safety, which can provide a reference basis for clinicians to determine the preferred treatment plan. The patient's curative effect is related to age, diabetes history, vascular infarction location, and intravenous thrombolysis time, which is helpful for clinicians to estimate the curative effect of patients, so as to appropriately modify the treatment plan of refractory patients.

## Figures and Tables

**Figure 1:** The incidence of bleeding between control group and observation group. ^*∗*^ indicates a significant difference (*P* < 0.05).

**Figure 2:** The incidence of MACE between control group and observation group. ^*∗*^ indicates a significant difference (*P* < 0.05).

**Table 1:** Comparison of vascular recanalization between the two groups (*n*, %).

Group	Number of cases	Complete recanalization	Recanalization	Vascular occlusion	Recanalization rate
Control group	50	18 (36.00%)	24 (48.00%)	8 (16.00%)	42 (84.00%)
Observation group	50	28 (56.00%)	20 (40.00%)	2 (4.00%)	48 (96.00%)
*χ*^2^ value					4.021
*P* value					0.045

**Table 2:** Comparison of the improvement of heart function between the two groups before and after treatment (*n*, mean ± SD).

Group	Number of cases	LVDs (mm)		LVEDD (mm)		LVEF (%)	
		Before treatment	After treatment	Before treatment	After treatment	Before treatment	After treatment
Controlgroup	50	47.24 ± 5.84	37.82 ± 6.15^*∗*^	54.73 ± 4.26	49.61 ± 3.84^*∗*^	43.04 ± 5.72	52.63 ± 6.08^*∗*^
Observation group	50	46.97 ± 5.46	34.14 ± 4.58^*∗*^	55.02 ± 4.38	45.43 ± 3.02^*∗*^	43.26 ± 5.16	60.18 ± 7.24^*∗*^
*t* value		0.239	4.815	0.336	6.051	0.202	5.647
*P* value		0.811	0.039	0.738	0.015	0.841	0.021

*Note.* Compared with the same group before treatment, ^*∗*^*P* < 0.05.

**Table 3:** Comparison of bleeding between the control group and observation group (*n*, %).

Group	Number of cases	Gum bleeding	Nasal mucosal bleeding	Gastrointestinal bleeding	Incidence
Control group	50	2	2	2	6 (12.00%)
Observation group	50	1	0	0	1 (2.00%)
*χ*^2^ value					3.895
*P* value					0.049

**Table 4:** Comparison of the incidence of MACE between the two groups (*n*, %).

Group	Number of cases	Heart failure	Angina pectoris	Arrhythmia	Recurrent myocardial infarction	Incidence
Control group	50	3	3	1	1	8 (16.00%)
Observation group	50	0	1	1	0	2 (4.00%)
*χ*^2^ value						4.012
*P* value						0.045

**Table 5:** Single factor analysis that affects the efficacy of patients after treatment (*n*, %).

Influencing factor		Number of cases	Reconnection group (*n* = 90)	Occlusion group (*n* = 10)	*χ*^2^ value	*P* value
Age	≥60 year	40	33 (36.67%)	7 (70.00%)	4.167	0.041
	<60 year	60	57 (63.33%)	3 (30.00%)		

Gender	Male	59	53 (58.89%)	6 (60.00%)	0.098	0.946
	Female	41	37 (41.11%)	4 (40.00%)		

Smoking history	Yes	45	37 (41.11%)	8 (80.00%)	5.512	0.021
	No	55	53 (58.89%)	2 (20.00%)		

Drinking history	Yes	43	39 (43.33%)	4 (40.00%)	0.142	0.832
	No	57	51 (56.67%)	6 (60.00%)		

History of diabetes	Yes	32	26 (28.89%)	6 (60.00%)	4.003	0.045
	No	68	64 (71.11%)	4 (40.00%)		

History of hypertension	Yes	38	34 (37.78%)	4 (40.00%)	0.986	0.891
	No	62	56 (62.22%)	6 (60.00%)		

History of myocardial infarction	Yes	22	17 (18.89%)	5 (50.00%)	5.076	0.024
	No	78	73 (81.11%)	5 (50.00%)		

Family history of coronary heart disease	Yes	18	16 (17.78%)	2 (20.00%)	0.125	0.862
	No	82	74 (82.22%)	8 (80.00%)		

Vascular infarction site	Anterior wall	46	49 (54.44%)	2 (20.00%)	4.273	0.038
	Inferior wall	54	41 (45.56%)	8 (80.00%)		

Intravenous thrombolysis time	≤2 h	58	56 (62.22%)	2 (20.00%)	6.586	0.014
	>2 h	42	34 (37.78%)	8 (80.00%)		

**Table 6:** Assignment for multivariate analysis of factors.

Factor	Variable	Assignment
Age	*X*1	<60 = 0, ≥60 = 1
Smoking history	*X*2	No = 0, yes = 1
History of diabetes	*X*3	No = 0, yes = 1
History of myocardial infarction	*X*4	No = 0, yes = 1
Vascular infarction site	*X*5	Anterior wall = 0, inferior wall = 1
Intravenous thrombolysis time	*X*6	≤2 h = 0, >2 h = 1

**Table 7:** Analysis of multiple factors affecting the efficacy of patients after treatment.

Influencing factor	*B*	SE	Walds	df	Sig.	Exp. (*B*)
Age	1.128	0.473	5.086	1	0.026	1.574
Smoking history	0.332	0.156	1.924	1	0.215	1.216
History of diabetes	1.306	0.512	4.864	1	0.032	2.089
History of myocardial infarction	0.415	0.192	2.158	1	0.174	1.236
Vascular infarction site	1.214	0.432	4.573	1	0.036	2.218
Intravenous thrombolysis time	1.294	0.465	5.315	1	0.022	2.308

## Data Availability

The data used during the current study are available from the corresponding author on reasonable request.
